The article "Volumetric Evaluations of Full-Arch Implant Supported Restorations and Their Role on Patients' Quality of Life: A Mixed-Model Analysis" was published in 2022. Journal: Biomed Res Int.

# Volumetric Evaluations of Full-Arch Implant Supported Restorations and Their Role on Patients' Quality of Life: A Mixed-Model Analysis

**DOI:** 10.1155/2022/3640435

**Published:** 2022-08-09

**Authors:** Ernesto Bruschi, Paolo De Angelis, Laura Papetti, Edoardo Rella, Giulio Gasparini, Antonio D'addona, Paolo Francesco Manicone

**Affiliations:** ^1^Private Practice, Frosinone, Italy; ^2^Department of Head and Neck and Sensory Organs, Division of Oral Surgery and Implantology, Fondazione Policlinico Universitario A. GemelliIRCCS—Università Cattolica del Sacro Cuore, Rome, Italy; ^3^Department of Head and Neck, Division of Oral and Maxillofacial Surgery, Fondazione Policlinico Universitario A. Gemelli IRCCS-Università Cattolica del Sacro Cuore, Rome, Italy

## Abstract

**Introduction:**

Full-arch, implant-supported hybrid restorations, employing tilted implants, can offer an efficient way of treating edentulous patients. Several factors, such as the timing of implant placement and the inclination of the fixture, can have a detrimental effect on their stability. This retrospective study is aimed at discerning the role played by those factors.

**Materials and Methods:**

Patients treated with full-arch, implant supported restorations were selected for this study; cone-beam computed tomography (CBCT) images, taken 3 months and 3 years after delivery of the final restoration, as well as peri-implant values, were obtained and compared; bone loss was measured on four sites for each implant and then averaged. These patients were recalled, and the OHIP-5 questionnaire was administered.

**Results:**

21 patients, with a mean age of 53 years, were included in the present analysis. 108 implants were placed, and 25 Toronto prostheses were delivered. According to a mixed-model analysis, tilted implants (0.51, *p* < 0.001) had a higher rate of bone loss, while implants placed in a healed ridge suffered less bone loss than immediate implants (-0.21, *p* < 0.001). Patient-level variables have a significant effect on this variable, as implants coming from the same subject share a similar risk of bone loss. The mean response to the self-administered OHIP-5 questionnaire was 1.53 ± 0.29; other variables did not have a statistically significant effect on this outcome. *Discussion/Conclusions*. The results of the present study show that Toronto bridges prostheses are an efficient procedure for treating edentulous patients, as their oral-related quality of life is reported as satisfactory even 7 years after delivery of the restoration. Tilted and immediate implants are more at risk of bone loss. Implants coming from the same subject share a similar risk of bone loss.

## 1. Introduction

While edentulism is a declining phenomenon, tooth loss remains, especially in underdeveloped countries, a major issue [1, 2], as edentate patients manifest a major impairment of their psychosocial functioning [3, 4] and suffer from great nutritional disturbances [5, 6].

Providing a prosthetic rehabilitation to these patients can notably improve many of their conditions [7].

Implant-supported restorations, given their stability and their appearance which mimics natural teeth, offer optimal results [8–10].

The conventional approach to implant therapy typically involves a two-step procedure where after implant placement, to achieve osseointegration, a healing time of variable length is allotted, and only after that, implants are loaded [11, 12]. Therefore, patients with failing dentition would need to go through a transitional period with a temporary denture [13]. The possibility of placing immediately loaded implants eliminates this occurrence and overall reduces the length of the procedure, offering a better psychological outcome [14–16].

Placing implants in a prosthetically favorable position that allows for the placement of a prosthesis with a favorable design is not always possible. While predictable outcomes may be obtained with surgical techniques available for augmenting bone in the maxilla or in the mandible [17, 18], patients may reject these more invasive procedures [19].

Another possibility to avoid advanced surgery, is to place tilted, longer, implants (between 30 and 45 degrees), increasing surface contact with the available native alveolar bone, while locating the implant platform in a position that may improve load distribution throughout the arch and reduce the length of the required cantilever [20, 21]. During the last decades, materials and techniques have improved continuously and immediate loading has revealed to be a predictable and reliable procedure, especially for full-arch rehabilitations [22–24].

The aim of this study was to evaluate the clinical outcomes and overall patients' oral-related quality of life with immediately loaded full-arch fixed prostheses supported by a combination of axial and tilted implants placed in postextractive sites or in healed sites and to compare the outcome of tilted versus axial fixtures in the same patients. The null hypothesis was that no difference in marginal bone level change would exist between axial and tilted implants placed in postextractive sites or in healed sites.

## 2. Materials and Method

This study is a retrospective, clinical review of patients treated at a private practice. A protocol was previously written and was then evaluated by the Ethical Committee of the Catholic University of the Sacred Heart and received ethical approval with code no. 3673.

All participants signed an informed consent for the prosthetic implant treatment and for participating in the present study.

All subjects treated with one or two implant supported, full arch restorations, between 2013 and 2014 were initially selected for the present study. Patients that were diabetic or that were defined as heavy smokers at the time of treatment were excluded. Similarly, patients without the required radiographical exams were excluded. These patients were recalled and invited to a follow-up appointment to assess the impact these prostheses had on their perceived quality of life; a self-administered questionnaire was therefore obtained. The OHIP-5 questionnaire was adopted [25] (Figure 1).

Patients that were unavailable (i.e., could not be recalled, did not want to attend the check-up) were also eliminated from the study.

### 2.1. Surgical Procedure

All patients had followed the hereby explained protocol.

Implant number, diameter, length, and position were planned based on clinical and radiographic analysis even though other factors, such as age and gender, patient opposing dentition, and bruxism were also considered.

All patients were submitted to a preoperative prophylaxis phase, where they received a supragingival scaling procedure and were instructed to rinse twice daily with a chlorhexidine digluconate 0.2% mouthwash starting 1 day before surgery and continuing for 7 days. Patients also received 2 grams of amoxicillin and clavulanic acid .(Augmentin, GlaxoSmithKline, Brentford, United Kingdom) 1 hour before surgery, while 2 grams/die were prescribed for the following 6 days.

All surgical procedures were performed under local anesthesia with articaine chlorohydrate and epinephrine 1 : 100,000. A mucoperiosteal flap was raised, and the initial cortical perforation with a round burn [2] was followed by osseous site preparation. Sequential drilling under copious saline irrigation was used to enlarge the implant bed.

Implants (Sweden & Martina SpA, Carrare, Italy) were placed according to the manufacturer's guidelines, and primary implant stability was achieved.

An implant-level impression was taken for the fabrication of a screw-retained, metal-reinforced, provisional restoration which was positioned the same day or within 24 hours. All centric and lateral contacts were assessed by a 40 *μ*m articulating paper (Bausch Arti-Check, Bausch Articulating Paper Inc., Everett Business Park, New Hampshire) and adjusted to check the rightness of both balanced occlusion and group function occlusion. The screw access was then filled with composite resin. Patients were scheduled for weekly control visits during the first month for tissue healing and prosthetic functionality assessment. After 3-4 months of loading, in the absence of complications, patients received the final restoration. A definitive impression of the arch was taken, and final acrylic restorations, reinforced with a metal framework with distal cantilevers of adequate posterior extension, were manufactured. All prosthetic restorations were made by the same dental technician.

At the completion of the prosthetic phase, implant and prosthetic conditions were evaluated by clinical examination and the occlusion was checked with occlusal papers of 16 and 8 microns (Hanel Shimstock Occlusion, Coltene Whaledent INC, Altstätten, Switzerland), and intraoral radiographs were carried out using the Rinn system to control distortion.

All patients were enrolled in a professional recall program for oral hygiene every 4 months.

All patients were recalled 3 months (*T*1) and 3 years (*T*2) after implant surgery, to assess the status of their rehabilitation. Moreover, a CBCT was taken at both time points to assess the status of the implants; these images were transferred into a dedicated software system (Ez3D-plus, VATECH Co. Ltd., Gyeonggi-do, South Korea) and analyzed by one designated examiner. The study used a 14-bit gray scale, a field of view (FOV) of 8 × 8 cm, voxel of 0.2 mm, and 15 s of exposure time. All radiographic and tomographic images were taken by the same operator [22].

At the same appointments, peri-implant values were measured with a periodontal probe (Periodontal Probe CP 15 North Carolina) (Hu-Friedy, Frankfurt Am Main, Germany) at 6 sites around each implant. All values were measured by the same calibrated examiner (*k* = 0.82). The periodontal probing depth at deepest site (PPDD) was used for the following analyses.

CBCT images taken 3 months and 3 years after delivery of the definitive rehabilitation from all patients included in the study were obtained, and from the sagittal and coronal images the distance between the implant neck at its crest module at, respectively, the mesial and distal bone level, and the buccal and oral bone level were measured.

The marginal bone level was then measured subtracting the value obtained at *T*2 from the value recorded at *T*1.

### 2.2. Outcomes

The primary outcome of the study was the analysis of peri-implant marginal bone loss, as measured at 4 sites (mesial, distal, vestibular, and oral). The marginal bone loss measured at 4 levels was then averaged to obtain a single value (MBLT (marginal bone level total)), used for the statistical analyses. The secondary outcomes were the analysis of the peri-implant parameters assessed at the 3-year follow-up, when compared to values recorded at the 3-month follow-up, and the self-administered questionnaire results, regarding the oral-related quality of life of these patients, obtained with the OHIP-5.

### 2.3. Statistical Analyses

Qualitative variables were described as absolute and percentage frequencies, while quantitative variables were summarized as mean and standard deviation.

To assess the relationship between the collected variables, which followed a normal distribution, and each outcome, multivariate mixed models were used, considering the implant as a statistical unit of reference, and including the prosthesis, these implants came from, nested in the patients these implants were placed, as random effect and all other variables (i.e., inclination, timing of placement, location, fixture diameter, fixture length, and sex) as fixed effect, with the MBLT, PPDD, and the OHIP-5 being the variables of interest.

All analyses were performed with STATA 17 (StataCorp. Stata StatisticalSoftware: release 17. College Station, Texas) a *p* value of <0.05 was set as the threshold for statistical significance.

## 3. Results

21 consecutive patients, 12 males and 9 females, with a terminal dentition in the upper or lower jaw rehabilitated with immediately loaded, screw-retained full-arch prostheses supported by axial and/or tilted implants placed in postextractive sites or in healed sites were included in this retrospective analysis.

The subjects had a mean age of 53 ± 10.2 years. 108 implants were placed.

17 patients received a single Toronto prosthesis (11 in the upper arch and 6 in the lower arch), while the remaining 4 received two prostheses. Of these 25 Toronto prostheses, 21 were supported by 4 implants, while the remaining 4 were supported by 6 implants. In 19 cases, implants were placed immediately after having extracted the remaining teeth, and in 6 cases, implants were placed in a fully healed alveolar process.

62 implants were positioned in the upper jaw, while 46 in the lower jaw. 56 implants were tilted (with an inclination of 30 to 45 degree), 76 implants had a diameter of 3.8 mm, while 32 had a diameter of 4.25 mm. 25 implants were 10 mm long, 14 were 11.5 mm long, 28 were 13 mm long and, finally, 41 were 15 mm long.

All prostheses were still in use at the last follow-up, and no implants were lost. The peri-implant status of included implants is reported in Table 1.

The final results of the multivariate mixed model (*N* = 108) are reported in Table 2; tilted implants had a higher rate of bone loss, with a coefficient of 0.49. This was statistically significant, even if only 4 tilted implants had a MBL higher than 2 mm.

Similarly, implants placed in a healed site had a reduced amount of bone loss, with a coefficient of -0.22, and this effect proved to be statistically significant. Therefore, postextractive implants had a significant higher average value.

In addition, the within subject and within prosthesis variability were significant in the previous model; therefore, implants coming from the same prosthesis tend to manifest similar values when compared to implants coming from a different one.

No one of the measured variables had a statistically significant effect on the PPDD (*N* = 108) (Table 3).

Overall, patients were appropriately satisfied with their implant-supported restorations, with a mean response to the OHIP-5 questionnaire of 1.53 ± 0.29; according to the included linear regression (Table 4), none of the included parameters had a significant effect on this variable (*N* = 17).

## 4. Discussion

The aim of this retrospective study was to evaluate and assess the clinical outcomes and the reliability of full-arch, implant supported restorations, comparing the effects of several variables. Simultaneously, the self-reported, oral-related quality of life of these patients was measured and compared.

According to our results, this type of rehabilitation is extremely reliable as no prosthesis was lost; this confirms the findings of other similar studies [26, 27].

Tilted implants are particularly efficient for rehabilitating patients with a fixed prosthesis, (Figures 2–4) even when anatomical contraindications are present; [28, 29] our mixed model results shows that tilted implants had a higher rate of marginal bone loss when compared to axially placed implants. In our sample, tilted implants were placed in the posterior region of the arch where (especially in the maxilla) bone quality is much lower and, usually, there is less bone available, making their positioning more challenging. Also, given their inclination, their platform is not positioned flush with the alveolar process but has an angle, creating an uneven zone of resorption along the crest module of the implant.

It must be pointed out although that we found a particularly small difference (0.38 mm) which might not be significant from a clinical viewpoint. Many articles available in the literature have stated the opposite [30, 31], but, to our knowledge, this is the first paper, together with one previously published by our group [32], that has observed the MBL on a CBCT analysis which provides an higher accuracy, when compared to bidimensional exams. Moreover, bidimensional exams can only offer an evaluation of the mesial and distal bone levels but cannot analyze the vestibular and the oral bone levels; meanwhile, a CBCT exam provides a tridimensional snapshot of the bone levels around the implant.

Immediately placed implants also had a higher rate of bone loss when compared to implants placed in a healed ridge; this confirms what other authors have said: postextractive implants have a higher risk of complications and a higher rate of bone resorption [33–35].

More so, implants coming from the same patient had similar amount of bone loss, and this concordance was found to be much more relevant than the effects of all the other variables; this is key as it shows that implant-level variables (such as position and inclination) have a marginal effect regarding peri-implant health when compared to patient-level characteristics (i.e., hygiene levels and prosthetic design). Again, this shows that for an implant-supported rehabilitation to be efficient and successful, adherence to a proper maintenance protocol is paramount.

Given the major interest that has been given in dentistry towards patient-centered outcome measures, one, if not the most relevant outcome of treating edentulous patients, is obviously the improvement of their quality of life, which can be measured with many different tools [36, 37].

Regarding these outcomes, measured in the present study with the OHIP-5, the included results demonstrate that this type of full-arch, implant-supported rehabilitation provides high satisfaction and is totally accepted by the patient. The number of implants and the timing of prostheses placement did not have a role in determining this variable.

These findings are obviously flawed by many biases, apart from the design of the study; the number of implants employed in each rehabilitation was not randomly defined but rather decided by the clinician, as well as length and diameter of each fixture. Also, it is possible that the patients who did not find their rehabilitation efficient, preferred to not participate in this study; therefore, making our results overestimated.

## 5. Conclusions

Tilted implants are an efficient solution for rehabilitating edentulous patients who would prefer to avoid more complex surgeries but have a slightly higher rate of bone resorption when compared to axial implants. Full-arch hybrid restorations provide a favorable outcome at a 3-year follow-up.

## Figures and Tables

**Figure 1:** The adopted version of the OHIP-5.

**Figure 2:** Panoramic X-ray images of an edentulous case treated with the protocol.

**Figure 3:** Typical case before (a) and after (b) treatment.

**Figure 4:** A CBCT image of one of the included cases.

**Table 1:** The peri-implant values of included implants (*N* = 108).

Variable		Mean	Standard deviation	95% confidence interval
Mesial MBL		2.11	0.07	1.97-2.25
Distal MBL		1.31	0.04	1.24-1.39
Vestibular MBL		1.11	0.02	1.06-1.15
Lingual MBL		0.99	0.02	0.95-1.02
Mean MBL		1.38	0.33	1.31-1.44
Mean PPDD		2.86	0.08	2.69-3.03

MBL: marginal bone level; PPDD: periodontal probing depth at deepest site.

**Table 2:** The results of the multivariate mixed model relative to marginal bone level total (MBLT) (*N* = 108).

	Coefficients	95% confidence interval	*p* value
Inclination			
Tilted implants	0.49	0.41-0.57	<0.001
Timing			
Implants placed in a healed site	-0.22	-0.35-0.09	<0.001
Position			
Lower arch	0.02	-0.04-0.09	0.97
Implant diameter			
4.25	0.35	-0.3–0.11	0.34
Implant length			
11.5	-0.17	-0.12–0.09	0.09
13	-0.32	-0.13–0.06	0.06
15	0.23	-0.8–0.13	0.13
Sex			
Female	0.02	-0.08-0.14	0.61

**Table 3:** The results of the multivariate mixed model relative to periodontal probing depth at deepest site (PPDD) (*N* = 108).

	Coefficients	95% confidence interval	*p* value
Inclination			
Tilted implants	0.38	0.09 - 0.67	0.21
Timing			
Immediate prostheses	-0.38	-0.81 0.18	0.215
Position			
Lower arch	-0.08	-0.5 0.33	0.69
Implant diameter			
4.25	0.12	-0.3 – 0.11	0.49
Implant length			
11.5	-0.48	-1.02 – 0.5	0.08
13	-0.73	-1.22 – 0.02	0.07
15	-0.59	-1.12 – 0.06	0.27
Sex			
Female	-0.01	-0.42 – 0.45	0.96

**Table 4:** The linear regression for the OHI-5 results (*N* = 17).

	Coefficients	95% confidence interval	*p* value
Timing			
Implants placed in a healed site	-0.04	-0.40-0.32	0.8
Position			
Lower arch	-0.28	-0.57-0.008	0.05
Sex			
Female	-0.14	-0.42-0.139	0.29

## Data Availability

The datasets used and/or analyzed during the current study are available from the corresponding author on reasonable request.
